# Application Effect of Meticulous Nursing on Community Elderly Patients with Coronary Heart Disease under the Background of Medical Treatment Partnerships

**DOI:** 10.1155/2021/3511985

**Published:** 2021-12-11

**Authors:** Wei Hao, Tian Ma, Chun Feng

**Affiliations:** ^1^Lvjing Community Health Service Center, Central Hospital Affiliated to Shandong First Medical University, Jinan Central Hospital Affiliated to Shandong University, Jinan 250013, Shandong Province, China; ^2^Health Care and Rehabilitation Ward, Jinan Municipal Hospital of Traditional Chinese Medicine, Jinan 250012, Shandong, China

## Abstract

**Objective:**

To explore the application effect of meticulous nursing on community elderly patients with coronary heart disease (CHD) under the background of medical treatment partnerships.

**Methods:**

A total of 96 elderly CHD patients treated in the community from July 2019 to July 2020 were selected as the research objects and divided into the experimental group (*n* = 48) and control group (*n* = 48) by the medical personnel according to their admission order. Clinical routine nursing was performed to the patients in the control group, and meticulous nursing under the background of medical treatment partnerships was conducted to the patients in the experimental group, so as to evaluate their quality of life (QOL) and self-care agency after intervention by the Chinese Questionnaire on Quality of Life in Patients with Cardiovascular Disease (CQQC) and Exercise of Self-Care Agency (ESCA) scale.

**Results:**

Compared with the control group after intervention, the patients in the experimental group presented significantly higher ESCA scores, HHI scores, and CQQC scores and longer 6 min walking distance (*P* < 0.001) and remarkably lower POMS scores (*P* < 0.001) and had obviously higher numbers of cases with various health-related actions (*P* < 0.05).

**Conclusion:**

Meticulous nursing under the background of medical treatment partnerships is a reliable method for improving the QOL and mood state of community elderly CHD patients, which greatly promotes patients' self-care agency and expectation. Further research will be conducive to establishing a better solution for patients.

## 1. Introduction

Coronary heart disease (CHD) is resulted from the narrowing or occlusion of the coronary artery lumen [1]. As a common cardiovascular disease (CVD), CHD places great pressure on healthcare systems in countries around the world. China Cardiovascular Diseases Report 2018 stated [2] that the number of CVD cases has reached 290 million, including about 11 million CHD patients, and the number of CHD cases and deaths will continuously show an upward trend in the next 5 years. Most CHD patients present with press and pain sensation in the middle piece segment of sternum or precordial region at onset, and severe cases may even develop sudden angina, radiating to the left dorsal shoulder and left upper extremity. CHD has a long duration, and its occurrence and progression are closely related to a variety of adverse behavioral habits. However, CHD patients have poor compliance in long-term treatment and avoiding adverse behavioral habits and often neglect the impact of adverse behaviors on the disease, thus leading to disease recurrence and aggravation that severely affect daily life. Therefore, a more systematic nursing intervention is needed to help patients relieve physiological symptoms and promote recovery [3]. Currently, traditional CHD care is still adopted in China, including following medical advice to implement nursing operations and health preaching, but clinical investigation found [4] that although traditional nursing intervention is basically able to meet the treatment needs, it lacks flexibility and pertinence and the emphasis on the emotions and psychology of patients, resulting in poor nursing outcomes [5, 6]. The concept of “medical treatment partnerships” was first proposed at the National Hygienical Conference in 2013 [7], which, through integrating different categories of medical institutions, establishing a well-defined and feasible mechanism for division of labor and cooperation, and improving the overall efficacy of the medical service system, aims to upgrade the service ability of the primary level and better achieve the purpose of graded diagnosis and treatment and satisfying the mass demands [8]. Meticulous nursing is a new type of patient-centered nursing model that develops corresponding nursing measures based on patient needs and focuses on details to finely process the contents of each nursing measure, thereby providing patients with better nursing services [9]. In this study, the effect of conducting meticulous nursing intervention under the background of medical treatment partnerships for community elderly CHD patients was explored to provide basis for clinical nursing.

## 2. Data and Methods

### 2.1. General Information

A total of 96 community elderly CHD patients treated in our hospital from July 2019 to July 2020 were selected as the study objects and divided into the experimental group (*n* = 48) and control group (*n* = 48) according to their admission order. The study met the World Medical Association Declaration of Helsinki (2013) [10]. Inclusion criteria: ① the patients met the diagnosis criteria for CHD in Guidelines for Diagnosis and Treatment of Coronary Heart Disease [11] and were diagnosed after coronary angiography, and their clinical symptoms included chest pain, shortness of breath, and chest compression; ② the patients were over 60 years old and conscious and had normal language communication ability; and ③ the patients and their family members understood the study and signed the informed consent. Exclusion criteria: ① the patients had combined malignant tumor; ② the patients had severe cerebrovascular disease; and ③ the patients were critically ill with acute myocardial infarction or grade IV cardiac function.

### 2.2. Methods

Drug therapy was performed to patients in the two groups to control condition progression and improve cardiac function, with the common drugs including aspirin, nitroglycerin, and nifedipine, and other measures such as oxygen inhalation were taken to support the treatment. Clinical routine nursing was carried out to the control group, including detection of vital signs, guidance on medication, prevention of complications, and conventional propaganda and education on disease [12].

Under the background of medical treatment partnerships and with the help of a sharing platform, meticulous nursing intervention was performed to CHD patients in the experimental group in the clinic. A total of 4 CHD management teams were established, and each team was consisted of 1 expert, 3 specialist nurses, and 1 community doctor and was responsible for 12 patients. The experts mainly participated in works such as training of community hospital and clinic and answering difficult problems, and the specialist nurses were responsible for implementing therapeutic lifestyle changes (TLC). In the early stage of treatment, the CHD management teams conducted the home visiting to patients at least once every 15 days, and after the patients' condition was stable, the frequency could be altered to once a month. For those with poor treatment effect, they should turn to the experts for diagnosis and treatment and establishing a “one-on-one” treatment regimen. A WeChat group was set up for the specialist nurses to share relevant CHD contents in the forms of voice messages, pictures, videos, and text messages at 10 o'clock every morning. During nursing intervention, condition monitoring was enhanced to focus on the condition changes, timely performing treatment and nursing, and effectively preventing complications. If the patients had dyspnea, symptomatic nursing should be adopted to ensure smooth breath, and the patients should keep in semireclining position under assistance, or in sitting position when necessary with both legs hanging down to reduce the returned blood volume. Psychological intervention was enhanced to encourage the patients to join more social activities, the psychological intervention skills such as “encouragement” and “implication” were emphasized to the patients' family members, timely attention was paid to the patients' emotional changes and psychological counseling was conducted, and the family members were encouraged to participate in the patients' recovery training. Patients did exercises under guidance; if they had breathing difficulties, exercises on sickbed were increased, such as stretching arms and swinging legs under assistance, with the training frequency being set reasonably according to their condition and physical ability, and when their breathing was improved, exercises at bedside or indoor exercises were carried out gradually, including march on the spot, walking, and squats, with the frequency and intensity increasing from low to high. The intervention time for both groups was 3 months.

### 2.3. Observation Indicators

The patients' self-care agency after intervention was evaluated by the Exercise of Self-Care Agency (ESCA) scale [13], which covered self-care agency, self-concept, self-care responsibility, and disease and health knowledge level. The total score of each dimension was 50 points, with higher scores indicating stronger self-care agency.

The mood state of patients in the two groups after nursing was evaluated by the Profile of Mood States (POMS) [14], which covered 7 dimensions, namely, fatigue, vigor, depression, confusion, anger, tension, and esteem-related emotions, and a total of 40 items. The total score was obtained by score for negative emotions and score for positive emotions, with higher scores indicating deeper mood state.

The 6 min walking distance of patients after intervention was measured, and the patients' expectation of improving their condition was evaluated by Herth Hope Index (HHI) [15], which covered relationship with others, attitude towards the present and the future, and the actions taken. The score range was 12–48 points, with higher scores indicating higher expectation.

The patients' QOL after intervention was evaluated by Chinese Questionnaire on Quality of Life in Patients with Cardiovascular Disease (CQQC) [16], including 6 items and 24 questions, such as physical strength, condition, medical service status, social psychological status, and work status. On a scale of 0–154 points, higher scores indicated better QOL.

The patients' compliance with health-related action was compared between the two groups, including regular reexamination, taking medicine according to medical advice, reasonable diet, and proper exercises. The numbers of cases compliant with health-related actions after intervention in both groups were counted.

### 2.4. Statistical Methods

In this study, the data processing was conducted with the professional statistic software SPSS24.0, the picture drawing software was GraphPad Prism 7 (GraphPad Software, San Diego, USA), the enumeration data were examined by *X*^2^ test and expressed by (*n* (%)), the measurement data were examined by *t*-test and expressed by mean ± SD, and differences were considered statistically significant at *P* < 0.05.

## 3. Results

### 3.1. Comparison of Clinical Data

The patients' clinical data including gender ratio, mean duration of disease, disease type, and residence status were not significantly different between the two groups (*P* > 0.05) and were comparable. See Table 1.

### 3.2. Comparison of ESCA Scores after Intervention

After intervention, the ESCA scores on various items of the patients in the experimental group were obviously higher than those in the control group (*P* < 0.001). See Table 2.

### 3.3. Comparison of POMS Scores after Intervention

After intervention, the POMS scores of patients in the experimental group were significantly lower than those in the control group (*P* < 0.001). See Figure 1.

### 3.4. Comparison of 6 Min Walking Distance and HHI Scores after Intervention

After intervention, the mean 6 min walking distance and mean HHI scores of the experimental group were significantly higher than those of the control group (*P* < 0.001). See Figure 2.

### 3.5. Comparison of CQQC Scores after Intervention

After intervention, the CQQC scores of the experimental group were significantly higher than those of the control group (*P* < 0.001). See Figure 3.

### 3.6. Comparison of Compliance with Health-Related Action after Intervention

After intervention, the numbers of cases with various health-related actions of the experimental group were significantly higher than those of the control group (*P* < 0.05). See Table 3.

## 4. Discussion

Research and investigations have found that there are 290 million patients with cardiovascular diseases in China and approximately 11 million of them suffer from CHD, which will lead to angina pectoris, heart rupture, cardiac embolism, etc., seriously threatening life safety [17]. Because of the long course of CHD, patients need to take medicine for a long time to maintain cardiac function while controlling predisposing factors and preventing complications in daily life to reduce the occurrence of adverse events such as sudden death and sudden myocardial ischemia [18]. Although conventional nursing provides good care for patients during their stay in the hospital, patients' dynamic condition when they are resting at home cannot be correctly grasped, leading to undesirable nursing effect. The selected cases in this study were the elderly CHD patients, and their decline of organ function due to the growth of age would bring about a series of complex clinical manifestations, and therefore, with all these nursing problems, the clinical nursing for them should be more comprehensive, systematic, scientific, and normative.

Generally, secondary and tertiary hospitals only can carry out short-term treatment for those with aggravation of CHD condition or severe complications, and rehabilitation treatment and health knowledge preaching after discharge still need to be completed by community hospitals [19, 20]. However, because of the current heavy load of diagnosis and treatment by specialists and the relative scarcity of medical and nursing resources in community hospitals, combined with the limited capacity of diagnosis and treatment service, there is a great need to explore a CHD management mode that is operational, propagable, and highly efficient to channel quality medical resources down to community level and optimize the contradiction between the number and quality of management, aiming to reduce the risk of disease recurrence and improve the quality of life [21]. The medical treatment partnerships model is effective in relieving bed pressure in secondary and above general hospitals by promoting the formation of a good medical order and widening referral channels and thus upgrading the rational configuration of medical resources [22]. A comprehensive community intervention study [23] implemented comprehensive intervention and follow-up visits to 527 patients with carotid atherosclerosis (CAS) and found that, after intervention, patients' awareness rate of risk factors for CAS and formation rate of health-related behaviors were significantly elevated than before, proving that the model of medical treatment partnerships could promote the quality of life in patients with chronic disease and improve their disease prognosis. In this study, meticulous nursing under the background of medical treatment partnerships was performed to the community elderly CHD patients, and through further analysis, it was found that compared with the control group after nursing intervention, the patients in the experimental group had significantly higher HHI scores and 6 min walking distance (*P* < 0.001) and obviously lower POMS scores (*P* < 0.001). Old age, long disease course, critical illness, and poor clinical prognosis bring many difficulties to clinical nursing for CHD patients. A foreign study demonstrated that [24] implementing meticulous nursing to elderly patients with CHD complicated with asthenia can effectively improve patients' asthenia condition and promote their quality of life. Meticulous nursing focuses on elaborateness and precision in the implementation process and pays more attention to the details of the work content, form, and process of nursing throughout all phases of nursing, so that it is more scientific, reasonable, and comprehensive, and through psychological intervention, limb rehabilitation, etc., patients' cardiac function is improved and their confidence to beat the disease is enhanced [25]. In addition, the study showed that after nursing intervention, the CQQC scores of the patients in the experimental group were significantly higher than those in the control group (*P* < 0.001), fully proving that implementing meticulous nursing under the model of medical treatment partnerships could effectively improve the QOL of CHD patients, which was of great importance for improving disease prognosis. Shortcomings of the study: CHD is a recurrent chronic disease with a recurrence rate, so long-term effects should be considered in clinical interventions. However, due to the limited duration of the study, long-term follow-up was not conducted, and therefore additional evaluation of long-term efficacy should be added to future studies; based on the limitation of the study area, the sample size enrolled in this study was only patients from our community, and the source of cases lacked diversity, so the conclusion obtained initially herein remains to be refined by more subsequent studies.

In conclusion, performing meticulous nursing intervention under the background of medical treatment partnerships is a reliable method to promote the self-care agency, improve the mood state, and upgrade the quality of life of community elderly CHD patients, and further study will be conducive to establishing a better solution for them.

## Figures and Tables

**Figure 1:** Between-group comparison of POMS scores after intervention (mean ± SD). Note: the horizontal axis denotes the experimental group and the control group, and the vertical axis denotes the POMS scores (points); after intervention, the POMS scores of the experimental group and the control group were (13.28 ± 3.17) and (19.87 ± 3.23), respectively; and ^*∗*^ indicates significant difference in POMS scores after intervention between the two groups (*t* = 10.088, *P* < 0.001).

**Figure 2:** Comparison of 6 min walking distance and HHI scores after intervention (mean ± SD). (a) The between-group comparison of 6 min walking distances after intervention; the horizontal axis denotes the experimental group and the control group, and the vertical axis denotes the distance in *m*; after intervention, the mean 6 min walking distances of the experimental group and the control group were (326.82 ± 18.36) and (273.24 ± 6.18), respectively; and ^*∗*^ indicates significant difference in the mean 6 min walking distances after intervention between the two groups (*t* = 19.162, *P* < 0.001). (b) The between-group comparison of HHI scores after intervention; the horizontal axis denotes the experimental group and the control group, and the vertical axis denotes the HHI scores (points); after intervention, the mean HHI scores of the experimental group and the control group were (37.99 ± 3.06) and (32.83 ± 2.77), respectively; and ^*∗∗*^ denotes significant difference in mean HHI scores after intervention between the two groups (*t* = 8.661, *P* < 0.001).

**Figure 3:** Between-group comparison of CQQC scores after intervention (mean ± SD). Note: the horizontal axis indicates the experimental group and the control group, and the vertical axis indicates the CQQC scores (points); after intervention, the CQQC scores of the experimental group and the control group after intervention were (127.84 ± 7.35) and (103.69 ± 6.67), respectively; and ^*∗*^ indicates significant difference in CQQC scores after intervention between the two groups (*t* = 16.858, *P* < 0.001).

**Table 1:** Between-group comparison of clinical data (*n* = 48).

Item	Experimental group	Control group	*X* ^2^/*t*	*P* value
Male/female	28/20	26/22	0.169	0.681
Mean duration of disease (mean ± SD, years)	4.25 ± 0.46	4.31 ± 0.51	0.605	0.547
Mean age (mean ± SD, years)	63.27 ± 3.46	63.32 ± 3.51	0.070	0.944
Disease type				
Myocardial infarction	14 (29.17)	12 (25.00)	0.113	0.737
Heart failure	18 (37.50)	15 (31.25)	0.416	0.519
Arrhythmia	7 (14.58)	9 (18.75)	0.300	0.584
Myocardial ischemia	9 (18.75)	12 (25.00)	0.549	0.459
Residence status				
Living alone	9 (18.75)	7 (14.58)	0.300	0.584
Living with family	24 (50.00)	26 (54.17)	0.167	0.683
Living in apartment for the aged	13 (27.08)	10 (20.83)	0.515	0.473
Others	2 (4.17)	5 (10.42)	1.387	0.239
Educational degree				
College	3 (6.25)	5 (10.42)	0.546	0.460
Middle school	15 (31.25)	14 (29.17)	0.049	0.824
Primary school	26 (54.17)	23 (47.92)	0.375	0.540
Untaught	4 (8.33)	6 (12.50)	0.447	0.504
Place of residence			0.379	0.538
Urban area	23 (47.92)	20 (41.67)		
Rural area	25 (52.08)	28 (58.33)		

**Table 2:** Comparison of ESCA scores after intervention (mean ± SD, points).

Group	Self-care ability	Self-concept	Self-care responsibility	Disease and health knowledge level
Experimental	42.17 ± 3.24	35.82 ± 4.27	42.33 ± 5.71	36.14 ± 5.64
Control	32.16 ± 3.26	28.47 ± 4.61	34.23 ± 5.26	29.26 ± 5.39
*t*	15.089	8.181	7.229	6.110
*P* value	<0.001	<0.001	<0.001	<0.001

**Table 3:** Comparison of compliance with health-related action after intervention (*n* (%)).

Group	Taking medicine according to medical advice	Reasonable diet	Regular reexamination	Proper exercises
Experimental	43 (89.58)	41 (85.42)	38 (79.17)	35 (72.92)
Control	29 (60.42)	32 (66.67)	29 (60.42)	25 (52.08)
*X* ^2^	10.889	4.631	4.002	4.444
*P* value	<0.05	<0.05	<0.05	<0.05

## Data Availability

The data that supported the findings of this study are available on reasonable request from the corresponding author.
